# Evaluation of Teaching Quality on IP Environment Driven by Multiple Values Theory Based on Big Data

This article has been retracted.

**DOI:** 10.1155/2022/4857155

**Published:** 2022-09-16

**Authors:** Xiujuan Gu

**Affiliations:** College of Marxism, Xiangtan University, Xiangtan 411105, China

## Abstract

Despite the fact that big data technology has been applied in education, there are no studies and cases that combine big data with ideological and political (IP) teaching quality. At the same time, the existing methods of IP teaching quality evaluation lack the consideration of multiple values, and the system is not complete and systematic. The use of big data analysis technology can improve the rigor of teaching quality assessment and make the data analysis more scientific, so as to improve the management system of universities and enhance the education quality. Therefore, this paper fully considers the background conditions of large data at this stage, on the basis of studying the methods of evaluating the quality of IP teaching in colleges. The big data about teaching quality is obtained by distributed algorithm, and multiple value indicators are drawn into the quality evaluation system as a main driver to emphasize the multiple value theory. Hierarchical analysis (AHP) method and fuzzy comprehensive evaluation (FCE) method are selected as the data analysis methods to provide evaluation basis for the proposed model. This model can further test the evaluation index system of education and further verify the rationality of the distribution of the weight of indicators at all levels. The evaluation results based on the large educational data and research data of a university show that the IP teaching quality of the university is excellent. The comprehensive evaluation model overcomes the limitations of traditional evaluation methods and provides a more comprehensive analysis about the teaching quality of IP teaching in colleges. Meanwhile, the conclusions obtained by the proposed evaluation model can be used for both the overall comprehensive evaluation of teachers' teaching quality and a single comprehensive evaluation of the single factor affecting teaching quality. Using the evaluation results obtained by the model, we can set up advanced models and encourage backward students to have evidence. With the single-index evaluation, we can know what advantages the IP teaching or a certain teacher has and what aspects need to be strengthened. Therefore, we can put forward reasonable suggestions to progress instructing strategies and educating quality.

## 1. Introduction

Big data refers to large information that cannot be captured, managed, processed, and organized in a reasonable amount of time by mainstream software tools to help businesses make more positive business decisions. Since 2012, the “big data” industry has been booming and has become a major topic of discussion in all sectors, including education [1]. Victor Mayer-Schönberger has made it clear that big data will reshape the education sector as a whole. Big data technology applied can help make more accurate decisions and enhance the creativity of colleges and universities [2]. Virtus has proposed a new approach to teaching that uses big data analytics to provide early warnings about student performance and improve academic outcomes [3]. Independent research in the U.S. argues that big data can overcome the reliance on traditional teaching methods on performance at the test stage by focusing on data on academic performance and learning paths for students [4]. By focusing on big data analysis, teachers are able to study academic learning by a more effective method. The application of big data in education can effectively help teachers adjust teaching schedules, enrich teaching resources, and allocate teaching weights [5]. Process evaluation analysis can be enhanced, and both teachers and students can grasp academic quality as a whole. In the investigation report issued by the U.S. Department of Education in 2012, the cases and areas of big data in U.S. education and the challenges faced were highlighted [6]. The report noted the ability of big data to capture never-before-seen threads in complex data, suggesting that big data in education has specific educational applications [7]. Therefore, the current teaching quality evaluation model can consider the introduction of big data technology to make the amount of data richer and the evaluation results more comprehensive.

Rapid update and development of big data analytical means provides a new platform and opportunity for college construction [8]. However, the quality of education, especially IP teaching, is experiencing new challenges. The purpose of IP teaching is to provide ideological guidance to educated people through a series of education. With the more advanced use of big data in the new era, educated people have broader channels to get new information, and at the same time, the impact of ponderous information has caused a certain degree of influence on educated people's thoughts [9]. To meet the need of development, ideological and political theory teaching must also make appropriate adjustments and innovations, integrate resources and technologies, and further realize its own development and innovation. The assessment of IP teaching quality is a prerequisite to guarantee the effectiveness of education. However, at present, two single indexes are considered in the traditional evaluation system of IP teaching equality, leading to the maladjustment on the needs of the current development of the era of big data [10, 11]. In the current ideological and political education quality evaluation system, due to the lack of standardized evaluation standards, the operation behavior of participants is not standardized, and the stratification between various information is not obvious, with a strong subjective consciousness. Therefore, it is a tremendous need to optimize the evaluation method of teaching quality and build a more evaluation system suitable for considering the big data on teaching equality [12, 13].

Values, as a part of social ideology, are the deep structure that governs the evaluation and choice of subjects [14]. Among them, the trend of value pluralism is inevitable. Compared with monistic values, plural values map out the complexity and differences of values, not just the certainty and uniformity of values. Pluralistic values refer to the existence of more than two values in society, in which one value has a dominant role and the other values have an influential role [15]. The influence of socioeconomic factors and diverse cultures has led to the simultaneous existence of multiple compound values in society, and these concepts show discrete, differentiated, and mutually dissolving states [16]. Influenced by economic globalization, various cultures, social trends, and values have emerged, causing profound changes in Chinese culture and values. Differences and a variety of values exist simultaneously in different countries, different fields, tradition and modernity, society, and the individual, breaking the single-value model and developing values toward the trend of pluralism, forming a pattern of multiple values coexisting [17]. The diversity and group nature of values are the basis for the occurrence of value pluralism at the current stage, while the sociohistorical nature and relative stability of values are the objective basis for the formation of core values at the current stage. Along with the improvement of education level and the deepening of the country's openness, values develop in a more diversified direction [18]. Therefore, the assessment of the quality of IP teaching at the current stage should also take the plurality of values into full consideration.

Both hierarchical analysis and fuzzy comprehensive judgment are good at dealing with imprecise and fuzzy information, simulating human comprehensive judgment and reasoning ability, and establishing a link between qualitative and quantitative analysis [19, 20]. Hierarchical analysis is good at expressing human subjective judgment in quantitative form [21]. It treats the study item as a system and makes decisions using the decomposition, comparison, judgment, and synthesis school of thought [22]. It provides an effective method for determining the weights of evaluation indexes in fuzzy evaluation. The fuzzy evaluation method has a strong comprehensive judgment ability, and the index weights determined by using hierarchical analysis method make the fuzzy evaluation more scientific [23, 24]. Fuzzy mathematics is a mathematical tool to study many problems with unclear boundaries in reality [25]. One of its basic concepts is fuzzy set, which can be used to comprehensively evaluate the problem [26, 27]. Fuzzy comprehensive evaluation is a method based on fuzzy mathematics and application of the principle of fuzzy relation synthesis to quantify some factors with unclear boundaries and difficult to quantify, so as to comprehensively evaluate the problem. This method has been applied in the evaluation of students' talents, graduate education evaluation, and other aspects [28].

Despite the fact that many colleges are using big data technology as a supplement to data analytics, there are no studies and cases of combining big data with IP teaching, while the existing IP teaching quality assessment methods lack consideration of multiple values and the system is not complete and systematic enough. Therefore, this paper fully considers the background conditions of big data at this stage and establishes an ideological and political teaching quality evaluation system driven by the theory of multiple values. In the evaluation model, the AHP analysis method and fuzzy mathematics theory are used to analyze the collected educational big data, so as to improve the reliability and effectiveness of the evaluation process and evaluation results. A case is selected for empirical analysis to verify the effectiveness of the evaluation method.

## 2. The Big Data Analysis in Teaching Equality Evaluation

### 2.1. Education Big Data and Collection

Educational big data has been applied in some colleges and universities in China, but some applications remain in the big data technology application layer rather than in the big data thinking application layer [29]. Hence, there are few application examples focusing on IP teaching. Big data platforms are created by many colleges in China, but basically, there is no big data platform for full-time research on IP teaching; some policy makers only consider big data as a tool for teaching assessment [30]. The big data platform can process data according to multiple information evaluations such as teachers' age, professional level, and teaching quality; analyze the impact of various characteristics on teaching quality; explore the potential relationship between various information; and mine more authentic evaluations.

Schools should be accountable to families, individuals, and society in general and satisfy demands of all students. A perfect teaching evaluation system can be built based on the big data analysis technology, and the opinions of various parties can be absorbed in a more standardized way, carry out the statistical work of information through a complete management system, and also use this technology to quickly identify the assessment for student quality by all parties and finally get a more accurate quality assessment report. Big data in education means all digital, text, image, audio, video, and other data generated in the education process, such as basic information of students, their academic test scores, activity tracks, learning behaviors and basic information of teachers, teaching designs, and lesson plans. These interrelated daily data are constantly gathered to form a massive data set with profound educational and teaching analysis value. Applying its big data to education will certainly bring about profound changes in educational philosophy, teaching methods, and evaluation systems. By mining and analyzing the data to find out the implied laws, it will provide a scientific basis for precise guidance of teaching and learning and educational decision-making, thus promoting educational transformation and quality improvement. The process and content of data collection is shown in Figure 1.

### 2.2. The Design of Data Mining

Data mining represents the process of mining implicit and valuable threads from massive complex information by means of algorithms [31]. The nature of data mining determines that the technology can contribute to the enhancement of instructing quality. It is not objective and fair, nor is it scientific, if a teacher is measured in teaching quality assessment only by assessing the appearance of data. In the whole data mining process, all factors affecting the evaluation results should be fully considered, the deeper reasons for the popularity or otherwise of teachers should be uncovered, the strengths and weaknesses of various types of teachers should be uncovered, and experiences and lessons should be drawn from them [32]. Hence, it is necessary to apply data mining technology in uncovering the deep knowledge hidden behind the data to provide school management with a reasonable basis for making decisions. In this study, data mining is chosen to extract the correlation data of teachers' teaching quality.

The most important setting in data mining is data association rules. Its technical principle is that there is some similarity between variables or data, and these data are interrelated. The method of association is to find the association information network between the data in the database by calculating the similarity between the data. Data mining association rules such as *M*⟶*N* style implication expressions set the dataset *D* = {*i*_1_, *i*_2_, ⋯*i*_*n*_} as the transaction dataset; *M* and *N* denote two subsets of the thing dataset *D* [33]. Moreover, *M*⟶*N* is measured by two metrics, namely, support and confidence. Additionally, *M*⟶*N* is measured by two metrics, i.e., support and confidence, and support, which means that the number of a certain item set present on the whole dataset is used to indicate the commonness of the rule on the dataset and thus determine the degree of rule association. Expressed as a percentage, the general formula is:

(1) $$\begin{array}{c} \text{support}\left(M⟶N\right)=\frac{P\left(M\cup N\right)}{DS}, \end{array}$$

where *DS* is the number of data sets.

The confidence level, on the other hand, indicates the probability that one transaction occurs in the presence of another transaction at the same time and is the main indicator for mining the main indicator of the association between data transactions, and the formula is

(2) $$\begin{array}{c} \text{confidence}\left(M⟶N\right)=\frac{P\left(M\cup N\right)}{P\left(M\right)}. \end{array}$$

To obtain an increase in the computational efficiency and reduce the computing time during the mining process, a minimum threshold is set. During the operation, as long as the error of the item set is less than the minimum threshold, the item set can be eliminated.

The algorithm of association rule mining is using the prior knowledge of frequent item sets to construct frequent item sets of all data sets by an iterative method of step-by-step search. The principle is to prune the item sets according to their support, as shown in Figure 2.

The implementation process of the algorithm is as follows:

1. Initially, the support of each item is determined by scanning the data set, and the frequent 1-item set of all item sets is obtained
2. Iteratively use the *k* − 1 item set obtained in the previous step to generate a new candidate *K* item set
3. In order to get the support of candidate items, the algorithm needs to scan the data set again
4. Calculate the support of candidates and delete candidate sets whose support is less than the lowest threshold
5. When no new frequent item sets are generated, the algorithm ends

In order to improve the efficiency of algorithm, the distributed algorithm is selected for data mining.

*n* arrange to confirm the effectiveness of the mining calculation; the evaluation data of all teachers in a university for the past five years were selected for the performance experimental comparison and analysis, as shown in Figure 3. Stand-alone operation refers to the frequent item set mining algorithm on one machine, which is characterized by small amount of data and low requirements for the memory size and computing performance of the machine. The mining task can be completed on one machine. The comparison found that when the data mining correlation analysis of the distributed algorithm was performed on the teachers' teaching process, when the data volume was small, the advantage of the stand-alone operation in running speed was more obvious, and when the data volume gradually increased, the advantage of the calculation rate of the distributed algorithm began to be obvious.

### 2.3. Data Analysis Methods

The cluster analysis is used for data analysis, which in essence is to divide the set of data objects into multiple parallel classes or clusters based on the similarity and dissimilarity between data, and finally the clusters are independent of each other, but the elements within the clusters have extremely high similarity. The specific algorithms of clustering include various, commonly used division-based, density-based, and network-based clustering algorithms. The density-based clustering analysis method is adopted in this paper. The characteristic is that it does not depend on distance but on density, which overcomes the disadvantage that the distance-based algorithm can only find “spherical” clusters. The core idea is that as long as the density of the midpoint in a region is greater than a certain threshold, it will be added to the similar clusters.

The basic process is:

1. First, each of the *n* samples of the data set is considered as the same class
2. Based on the similarity distance calculation
3. Select the sample with the greatest similarity as a class
4. Then, select the next most similar samples as a class, and so on, and so forth, and continue the operation

The similarity distance calculation method used in the calculation process is as follows:

(3) $$\begin{array}{c} \text{dist}\left(p\right)={\left(\overset{n}{\underset{i=1}{\sum }}{\left|x_{i}-y_{i}\right|}^{p}\right)}^{1/p}. \end{array}$$

When *p* = 1, it is called Euclidean distance:

(4) $$\begin{array}{c} \text{dist}\left(1\right)=\left(\overset{n}{\underset{i=1}{\sum }}\left|x_{i}-y_{i}\right|\right). \end{array}$$

When *p* = 2, it is called the Manhattan distance.

(5) $$\begin{array}{c} \text{dist}\left(p\right)={\left(\overset{n}{\underset{i=1}{\sum }}{\left|x_{i}-y_{i}\right|}^{2}\right)}^{1/2} \end{array}$$

When *p* tends to infinity, it is called the Chebyshev distance, at which point

(6) $$\begin{array}{c} \text{dist}\left(p\right)={\left(M\text{ax}\left|x_{i}-y_{i}\right|\right)}^{p}. \end{array}$$

Where the relative entropy distance is calculated using the following equation.

(7) $$\begin{array}{c} D\left(\left.p\right|\left|q\right.\right)=\frac{2}{1-a^{2}}\left(1-\int p{\left(x\right)}^{\left(1+a\right)/2}q{\left(x\right)}^{\left(1-a\right)/2}dx\right). \end{array}$$

## 3. The Establishment of IP Teaching Quality Assessment System

### 3.1. The Need for Multiple-Value Theory Drive

First of all, students have strong plasticity and are in the important period of cultivating correct values and outlook on life. However, in the loose college management environment, coupled with the popularity of network information tools, it is troublesome to maintain a strategic distance from the effect of various ideas. Although college students have certain self-discipline and the ability to distinguish right from wrong, their ideological and moral concepts will eventually be slightly shaken in the face of complicated information and ideas. In today's new environment, the value orientation of college students presents a pluralistic status quo, and this phenomenon should attract the attention of the IP teaching. In today's rapidly developing social era, people's ideology and social value system are experiencing great challenges, and values for college students in the development stage are changing constantly, and such values are often related to the views on society and the future; especially in the pluralistic environment, focusing on the pluralistic values of contemporary students has gotten to be an critical assignment of political instruction work. After opening up, ideas and society are progressing together, and there are more and more exchanges between Chinese and Western cultures, so diversified ideas and cultures are inevitable. The pluralistic characteristics of contemporary college students' values are related to the diversified social pattern composed of diversified subjects, which makes the life of social phenomena colorful, but may also cause confusion of thoughts and social disorder. It should be noted that in the pluralistic pattern of contemporary students' values, healthy and upward values are still dominant, but the influence of pluralistic values should be paid attention in the quality assessment of IP teaching, and the IP teaching assessment system driven by the theory of pluralistic values should be established.

### 3.2. Analysis Methods

Since teaching assessment subjects are an important aspect of conducting student teaching quality assessment, more subjects should be covered to enrich the final teaching quality assessment data [34]. However, in the context of big data, the dramatic increase in the number of subjects inevitably leads to the complexity of the model and the inefficiency of the computation [35]. Therefore, in order to avoid mutual interference between calculations and optimize the hierarchical structure among data sets, AHP and FCE methods are selected to study education big data.

The fundamental rule of AHP is to treat the complex issue beneath ponder as an expansive framework and to sort out the deliberate pecking order of the interaction between the variable interior of the framework by analyzing different component interiors of the framework. When applying the hierarchical analysis method to analyze the decision problem, the problem is firstly hierarchized, and the complex problem is decomposed into a collection of multiple levels of elements reached by attributes and connections to achieve the purpose of constructing a hierarchical structural model. In general, these levels can be divided into the top, middle, and bottom levels as shown in Figure 4.

To provide more credible data, pairwise comparison matrices were established for the factors. The errors and compatibility are based on the analysis of consistency indicators.

The consistency indicators were calculated using the following formula.

(8) $$\begin{array}{c} C.I=\frac{\lambda_{\max}-n}{n-1}. \end{array}$$

Consistency ratios are

(9) $$\begin{array}{c} C.R=\frac{C.I}{R.I}. \end{array}$$

Routinely, if the *C*.*R* judgment matrix is a consistency matrix, the consistency value calculated according to it is acceptable; otherwise, the judgment matrix has to be remodified. The consistency test is performed on the calculated total ranking of the stratum indexes, and all levels are gradually performed from the higher to lower levels. Let the judgment matrix of each relative comparison of the elements in and related to the criterion layer be tested for consistency in the final single ranking test, and the consistency hierarchical index *C*.*I*(*j*), (*j* = 1, ⋯, *m*) of the single ranking is derived, whose corresponding average randomly selected consistency indicators are derived in the hierarchical single sort, and the final total sorted random consistency ratio is

(10) $$\begin{array}{c} C.R=\frac{\sum_{j=1}^{m}C.I\left(j\right)a_{j}}{\sum_{i=1}^{m}R.I\left(j\right)a_{i}}. \end{array}$$

When *C*.*R* < 0.1, the total hierarchical ranking results can be considered consistent.

The FCE method is also a fuzzy mathematical algorithm established in the evaluation process to quantify and synthesize the nonlinear evaluation in reality and finally get comparable quantitative results. The comprehensive evaluation of education big data using the fuzzy mathematical method will also be closer to the real situation. Its main evaluation steps are as follows.

1. Calculate the assessment index of the FCE object

(11) $$\begin{array}{c} U=\left\{u_{1},u_{2},\cdots \cdots ,u_{p}\right\}. \end{array}$$

(2) Calculate the subject's rubric level domain

(12) $$\begin{array}{c} V=\left\{v_{1},v_{2},\cdots \cdots ,v_{p}\right\}. \end{array}$$

(3) Establish the fuzzy affiliation matrix *R*

After establishing the fuzzy subset of the rank, we must gradually quantify each factor *ui* of the selected evaluation object, determine the affiliation matrix of the fuzzy subset of the evaluated object, and then obtain the fuzzy relationship matrix of the evaluated object:

(13) $$\begin{array}{c} R={\left[\begin{array}{c} r_{11}r_{11}\cdots r_{1m}\\ r_{21}r_{22}\cdots r_{2m}\\ \cdots \cdots \cdots \cdots \\ r_{p1}r_{p2}\cdots r_{pm} \end{array}\right]}_{pm}. \end{array}$$

(4) Determine the weight vector *w* of evaluation factors

In fuzzy comprehensive evaluation, the analytic hierarchy process is used to determine the weight vector of evaluation factors *W* = (*w*_1_, *w*_2_, ⋯, *w*_*n*_, ). The analytic hierarchy process determines the relative importance of each factor, so as to determine the weight coefficient and normalize it before synthesis.

(5) Synthesize the evaluation result vector of FCE

Using a suitable weight set to synthesize the affiliation matrix with each evaluated thing, the evaluation result vector of this evaluated object can be obtained, namely.

(14) $$\begin{array}{c} K\cdot R=\left(a_{1},a_{2},\cdots ,a_{p}\right){\left[\begin{array}{cccc} r_{11} & r_{11} & \cdots & r_{1m}\\ r_{21} & r_{22} & \cdots & r_{2m}\\ \cdots & \cdots & \cdots & \cdots \\ r_{p1} & r_{p2} & \cdots & r_{pm} \end{array}\right]}_{pm}=S. \end{array}$$

(6) Analysis of the FCE result vector

We use the weighted average to determine the subordinate rank. The multiple evaluated objects can be used to calculate their corresponding scores.

### 3.3. Introduction of Indicators

The assessment of IP teaching quality in colleges and universities should not only absorb the opinions of students and teachers in the school but also consider the opinions of government authorities on the school, mutual evaluation between teachers and students, and social evaluation. This paper constructs an index system of IP teaching assessment from five aspects: school management quality, teaching preparation, students' multiple values, teaching resources, and academic quality.

School management quality: It is the guarantee of the normal operation of school education and teaching. Only the normal operation of school management mechanism can make teachers complete teaching tasks efficiently.

Teaching preparation: There are many uncertain factors in the course of teaching, which have a certain impact on the smooth implementation of teaching. Adequate teaching preparation is an important guarantee for the teaching quality of the course. Therefore, teaching preparation is an important indicator to measure the teaching quality.

Students' multiple values: From the background of the development of the current era, it is necessary to enhance the effectiveness and guidance of the study of multiple values, so students' different values should be included in the evaluation content.

Teaching resources: Rational use of teaching resources is an important means of auxiliary teaching. In addition, the use of teaching resources can create a richer and interesting learning environment for students and enhance their interest in learning. Therefore, teaching resources are an indispensable part of teaching quality evaluation.

Academic quality: Academic quality is an important reflection of teaching effect and feedback on the completion of teaching objectives. In the teaching process, through the examination of students' studies, we can improve students' participation and attention, so as to ensure the realization of teaching goals.

It contains 5 primary indicators and 18 secondary indicators, as shown in Table 1.

## 4. Teaching Quality Assessment and Analysis

### 4.1. Data Sources and Weighting Determination

Through the online learning platform and the school's educational administration system, teachers' teaching preparation, students' examination results, online learning, attendance, and so on are collected. Based on the big data mining means, the information of teaching cases, students' performance, postclass feedback, and school management uploaded by teachers in the teaching platform was mined to provide reference for the content of indexes B1, B2, B4, and B5 parts. At the same time then, questionnaires were designed for all students and teachers of a Chinese university, respectively, and research on teaching quality as well as students' behavior was conducted to provide reference for the calculation of indexes B3 and B5. Finally, the reliability and validity of the evaluation indexes were tested by questionnaires for the teachers of civic education, and the satisfaction survey of the constructed civic education teaching evaluation index system was conducted, and the results are shown in Figure 5.

Based on the evaluation of the feedback, a two-by-two comparison of each index at the same level in Table 1 was conducted to construct a judgment matrix for the two-by-two comparison and finally a consistency test. Taking the B-C level as an example, the judgment matrix and its processing results were obtained, as shown in Figure 6.

From the processing results, we can further obtain the relative weight vector *W*0 and the maximum eigenvalue *λ*_max_ normalized at the B-C level as *W*0 = [0.33, 0.07, 0.43], respectively. *W*2 = [0.28, 0.18, 0.45, 0.47], *W*3 = [0.44, 0.28, 0.30, 0.25], *W*4 = [0.41, 0.34, 0.68], *W*5 = [0.54, 0.27, 0.21, 0.13], and *λ*_max_ = 5.887.

The consistency test is performed on the judgment matrix of Figure 5, and the average value of the consistency index RI = 1.43 is obtained by querying the average random consistency index table, and then, the consistency ratio CR is calculated to be 0.004 according to the calculation formula of the consistency index. Because the value is less than 0.1, the consistency test of the judgment matrix passes.

The consistency of the secondary indicators is judged as follows:

Judgment of “School management quality”: *λ*_Max_ = 4.0231, CI = 0.0034, CR = 0.0045 < 0.10, passed the consistency test;

Judgment of “Teaching preparation”: *λ*_Max_ = 4.1345, CR = 0.0028, CR = 0.0031 < 0.10, passed the consistency test;

Judgment of “Student diversity values”: *λ*_Max_ = 4.2378, CR = 0.0056, CR = 0.0051 < 0.10, passed the consistency test;

Judgment of “Teaching resources”: *λ*_Max_ = 4.0891, CR = 0.0032, CR = 0.0071 < 0.25, passed the consistency test;

Judgment of “Academic quality”: *λ*_Max_ = 4.4329, CR = 0.0033, CR = 0.0021 < 0.10, passed the consistency test;

### 4.2. Quantitative Assessment of Teaching Quality

Based on the statistical results, the proportion of each evaluation level is calculated. Among them, the evaluation set *E* = excellent, good, medium, poor, bad good, medium, poor, bad, and assign values to the evaluation set and establish the weights of the IP teaching quality evaluation system as shown in Figure 7.

Taking “teaching preparation” as an example, according to the results of IP teaching quality evaluation, its affiliation matrix can be obtained as

(15) $$\begin{array}{c} R_{3}=\left[\begin{array}{c} 0.060.420.520.000.00\\ 0.330.380.160.010.12\\ 0.340.240.060.320.04\\ 0.770.040.060.010.12 \end{array}\right]. \end{array}$$

On this basis, the ultimate assessment comes about for educating and learning quality of the university's IP teaching (the second level of FCE), expressed in terms of affiliation, can be obtained as follows: *p* = (0.51, 0.11, 0.30, 0.05, 0.03). (0.11, 0.30, 0.05, 0.03). “poor,” and 3% “poor.” According to the principle of maximum affiliation, in the five levels of “excellent, good, moderate, poor, and bad,” we have 0.51 > 0.11 > 0.30 > 0.05 > 0.03. Therefore, the overall assessment of the quality of the university's ideological and political courses is “excellent.” After the investigation and analysis, the university's ideology course has been offered for a long time, and the teachers of the course are experienced in the selection of online resources. At the same time, the university's faculty team is reasonably constructed, and the interaction rate between teachers and students is high, so the overall teaching quality of civic education is excellent.

Also, based on this assessment model, the objective evaluation results can be visualized based on the traditional geometric method. For example, Figure 8 shows a schematic diagram of the fuzzy evaluation structure of IP teaching quality of two different teachers; it can be clearly found that teacher B has better teaching quality of the course and teacher A needs to strengthen teaching preparation and pay consideration to the scholastic quality of understudies.

The integration of qualitative and quantitative analyses is one of the advantages of this evaluation model. This paper describes the subjective issues within the assessment of teaching quality with scientific quantitative means. Through FCE, it is reduced to the quantitative expression of evaluation grade and each price index, which makes the qualitative analysis and quantitative analysis better integrated and overcomes the subjective randomness in the evaluation of teachers' classroom teaching quality. At the same time, the conclusion obtained by the AHP method can not only carry out the overall comprehensive evaluation of teachers' teaching quality but also make a single comprehensive evaluation of a single factor affecting teachers' classroom teaching quality. Using the results of the comprehensive evaluation of classroom teaching quality, we can establish advanced models and motivate the underachievers. Using single index evaluation, we can know what advantages IP teaching or a teacher has and what aspects need to be strengthened, so as to put forward reasonable suggestions to progress instructing strategies and educating quality. Based on the proposed evaluation model, the teaching quality of college students can be compared and analyzed, and the advantages and disadvantages of cultivating talents between schools can be found, and an objective evaluation can be given. At the same time, with the help of big data technology, we can find relevant information in time when talents are introduced, which also plays a certain role in supervising the teaching quality evaluation of colleges and universities, making the teaching quality evaluation transparent.

## 5. Conclusion

Based on the study of teaching quality assessment methods of IP teaching, the paper combines the background of big data and mines education data through big data technology. Multivariate value indicators are introduced, and a comprehensive evaluation model to assess the teaching quality of IP teaching based on AHP hierarchical analysis and fuzzy comprehensive evaluation method. The main conclusions are as follows:

1. The rise of big data innovation has advanced information-based education and has enhanced the IP teaching in colleges. Big data has improved the carrier of ideological teaching and moved forward the environment of ideological instruction. Agreeing to the investigation and preparing work of big data, it can be utilized with the Web and its portable terminal, so as to way better meet the learning needs of understudies and advance the improvement of high quality and high effectiveness of ideological teaching in colleges.

2. In the pluralistic pattern of contemporary students' values, healthy and upward values are still dominant, but the influence of pluralistic values should be paid attention in the quality assessment of IP teaching, and a IP teaching assessment system driven by the theory of pluralistic values should be established.

3. From the factors affecting teaching quality, it should be most appropriate to develop a more suitable evaluation index system for IP teaching from four aspects: school management quality, teaching preparation, students' multiple values, teaching resources, and academic quality.

4. A teaching quality assessment model based on AHP is constructed, which can further test the education evaluation index system and can deeply verify the rationality of the distribution of weights of indicators at all levels. The evaluation results obtained from a university based on the educational data and research data show that the IP teaching quality is excellent. It has certain applicability to the construction of evaluation system for similar research objects.

## Figures and Tables

**Figure 1:** The process and content of data collection.

**Figure 2:** The principle is to prune the item sets.

**Figure 3:** The performance experimental comparison and analysis.

**Figure 4:** The top, middle, and bottom levels of a hierarchical structural model.

**Figure 5:** The satisfaction survey of the constructed civic education teaching evaluation index system.

**Figure 6:** The judgment matrix of the B-C levels.

**Figure 7:** The weights of the IP teaching quality evaluation system.

**Figure 8:** A schematic diagram of the fuzzy evaluation structure of IP teaching quality of two different teachers.

**Table 1:** The primary indicators and secondary indicators used in the IP teaching assessment.

Main object	Primary indicators	Secondary indicators
Quality of IP teaching (A)	School management quality (B1)	Faculty composition (C11)
		Teaching environment (C12)
		Teaching conditions (C13)
	Teaching preparation (B2)	Preparation for class (C21)
		Emergency preparedness (C22)
		Proficiency in teaching tools (C23)
		Mobilization of students (C24)
	Student diversity values (B3)	Honest and trustworthy (C31)
		Love working (C32)
		Willingness to help (C33)
		Sense of collective honor (C34)
	Teaching resources (B4)	Video material (C41)
		Case resources(C42)
		Test resources (C43)
	Academic quality (B5)	Academic performance statistics analysis indicators (C51)
		Teaching interaction rate (C52)
		Student satisfaction (C53)
		Homework completion (C54)

## Data Availability

The datasets used during the current study are available from the corresponding author on reasonable request.
